This article has been retracted.

# Exploring Wavelet Transform-Based Image Enhancement Algorithm for Image Restoration of Long March National Cultural Park

**DOI:** 10.1155/2022/1434763

**Published:** 2022-06-29

**Authors:** Ruiming Wang

**Affiliations:** Shaanxi Normal University Academy of Fine Arts, Beijing 710061, China

## Abstract

China has taken the lead in exploring the construction of large-scale public cultural parks. By restoring the relics of the Long March, we can further promote the spirit of the Red Army, inherit the red gene, contribute to national pride, and contribute to local economic development. A new community will be built with culture, education, tourism, and leisure as the main contents. System aberration, human interference, motion, and system noise can all lead to image quality degradation. Wavelet enhancement technique is to use Wiener filtering in the Fourier region, using other properties of wavelets for filtering. The wavelet analysis method was used to recover the images within the Long March National Park, and the corresponding processing was carried out to achieve a better recovery effect. Through comparative tests, it was found that the algorithm had an average reduction of 223 iterations and an average increase of 11.264 in signal-to-noise ratio when iterating, and the number of iterations was also greatly improved. The higher the wavelet coefficients are, the higher the noise is. This paper introduces a new wavelet transform-based image restoration technique for national parks.

## 1. Introduction

The Chinese government has issued a programme for the construction of the Great Wall, the Grand Canal, and the National Long March National Cultural Park, as well as adequate preparations for the Great Wall, Grand Canal, and Long March National Cultural Park strategies [1]. As a result, the question of how to restore the national cultural center's image has become a focus of attention [2]. Scholars have also worked on the theoretical origins, development path of cultural and tourism integration, and main drivers of management system and policy innovation in order to provide a theoretical foundation for the construction of China's Long March National Cultural Park [3]. The transmission, conversion, transfer, and display of images in various image recovery systems can result in image quality degradation, which is primarily manifested by image blurring, distortion, and noise [4]. Image enhancement can be selectively enhanced according to the actual situation in the case of uninteresting images without investigating the causes of deterioration [5].

People's lives have been greatly improved by the development of information processing, computer, and communication technologies, while social needs are a major driving force behind technological advancement [6]. Fast processing speed, large information capacity, and high resolution are all advantages of optical image processing technology [7–9]. Due to processing accuracy, poor stability, and inconvenient equipment operation, it is less flexible than digital image processing for all types of requirements, and it is constrained by the actual production process and equipment materials. Wavelet analysis methods have a better recovery effect because the wavelet transformed image structure and texture have different resolutions. The wavelet transform is a multiscale component that can be processed in minute details using time and space domain sampling steps corresponding to different size components [10].

Single resolution image processing and analysis is no longer suitable for practical needs [11]. Wavelet analysis is a new time-frequency analysis technique [12]. It is based on the traditional FFT analysis method, which has practical value in practice and a great theoretical breakthrough [13]. Imaging events, such as regions and lines, are interesting and often occur at different spatial scales [14]. The ecological environment of the 15 provinces along the Long March has been better protected and restored, cultural tourism bases have been basically built, and the coordinated development of cultural tourism and cultural tourism has matured [15]. Imagery is an image that simulates and describes the similarities of objective things, and it is both a reflection of objective existence and a human mental activity. The study of wavelet transform for image reconstruction is of great value for both theoretical and military and civilian applications. This paper has several innovative features as follows.

1. The wavelet transform image enhancement method is a guideline for image restoration within Changting National Park.
2. The wavelet transform method is used to study the image restoration within the Long March Park and the restoration of the Long March Park.
3. Taking the histogram transformation of the image restoration of Long March Park as the basic idea, the wavelet transform was used to improve the image restoration of Long March Park.

## 2. Related Work

### 2.1. Image Restoration of Long March National Cultural Park

Long March cultural tourism resources are rich in variety, widely distributed, unique in theme and profound in connotation, with historical and cultural relics, residences of former generals and activists, and important battlefields. And clear, high-quality images are required in many applications. There are correlations and differences between network interests and tourism footfall networks, and on this basis, red tourism development potential areas such as Xiangzhong, Qianchuan, northern Shaanxi, and other key red tourism areas are identified. Therefore, the image restoration of the Long March National Cultural Park has led to increasing expectations for corresponding digital image processing technologies.

Pardhasaradhi et al. directly used the degraded system function that causes image degradation as prior knowledge and calculated the inverse permutation function of this function to recover the blurred image without considering the noise factor that forms the blurred image [16]. Ashwini proposed a multi-frame Wiener filtering method to address spatial and temporal correlation, which is a new development in Wiener filtering in recent years [17]. Kannoth and Kumar used an inverse filtering reconstruction algorithm to obtain relatively accurate reconstructed images, but noise often occurs in practical problems and the reconstructed images obtained using the inverse filtering algorithm are not effective [18]. Subramaniam et al. explicitly proposed a recursive filtering algorithm that can better suppress noise, reduce ringing, and achieve better blind image reconstruction under low conditions [19]. Pullagura et al. proposed a novel method for motion blur image reconstruction that overcomes the decision of the inverse convolution reconstruction algorithm, which is the concept of using statistical information from the image and noise to select the transform function that minimizes the mean square error [20].

Image restoration of the Long March National Cultural Park should be based on the main red tourism resources, and the development strategy of classification policy, segmentation development, and shortage remediation should be implemented. Existing scholars have conducted long-term research on image restoration technology and achieved many research results, but there are still many problems that need to be improved in order to meet the demand for more perfect image restoration.

### 2.2. Wavelet Transform Image Enhancement Algorithm

Wavelet analysis is a storage mapping file technique applied to large images. The culture of Chinese excellent traditional culture, revolutionary culture, advanced socialist culture, and other cultures are organically integrated into cultural tourism, penetrating into the heart of every person, and inspiring the universality and self-confidence of culture from the deepest level of the heart. Different enhancement methods have their own characteristics, and a single enhancement algorithm cannot improve the overall enhancement effect.

Arunachalaperumal and Dhilipkumar fleshed out the spatial concept of wavelet transform and combined multiple theories of wavelets, which led to a great improvement in the time-frequency characteristics of wavelet analysis [21]. Nazeeburrehman and Hussain proposed a global histogram equalization algorithm based on local features [22]. Currently, image enhancement techniques mostly use both linear and nonlinear approaches. Chen and Guo argued that multilayer grayscale distributions have complex properties that lead to many uncertainties, inaccuracies, and other problems [23]. Thus, fuzzy set theory can be used for the image processing. Anand proposed a new method for reducing wavelet thresholds and obtained an optimal proof from an asymptotic point of view [24]. Mehra et al. is mainly engaged in image modeling, image decomposition, wavelet transform, and image decomposition [25].

Wavelet image enhancement techniques enable local transformation of images, including spatial pixels and transformed areas.

## 3. Image Enhancement Algorithm

### 3.1. Gray Scale Transformation in Park Image Restoration of the Long March

Image restoration in national cultural parks is of great practical significance in enhancing national cultural confidence, demonstrating the long-term influence of excellent Chinese culture, and enhancing the charm of red culture [26]. Long March cultural tourism resources are closely related to natural ecology, history and culture, and ethnic culture, and have strong attraction and development potential [27]. Therefore, it is necessary to restore the images for the purpose of reducing noise and improving the image quality. By changing the gray scale, the contrast of the image can be improved, thus enhancing the clarity and prominence of the image. Wavelet analysis for image fusion is used for noise reduction processing as shown in Figure 1.

First, in order to highlight the target of interest in the image, the gray details of the feature objects are stretched and the uninteresting gray levels are suppressed as needed. Therefore, if both time and frequency domain resolution are to be improved, the wavelet master function must be selected appropriately. The gray levels of the original image are listed and the total number of occurrences of each gray level is calculated. Calculate the gray level histogram of the original image according to the following equation:

(1) $$\begin{array}{c} p\left(r_{i}\right)=\frac{n_{i}}{N}\left(i=0,1.2,\ldots ,300\right). \end{array}$$

*r*_*i*_—Grey level, *n*_*i*_—Total number of occurrences of gray levels, *N*—Total number of original image pixels, *p*(*r*_*i*_)—Probability of occurrence of gray scale.

The member function is called to calculate the *x* coordinate of the intersection point, and the *z* coordinate of the intersection point must be the height of the current sublevel, so there is no need to calculate the *z* coordinate of the knife position point without interference above this point:

(2) $$\begin{array}{c} z{}^{\prime }=\text{MAXINUM}\left\{z\left(i,j\right)+h\left(i,j,m,n\right)\right\}. \end{array}$$

*h*(*i*, *j*, *m*, *n*)—Height of contact *z*(*i*, *j*) to center point.

Wavelet transform is first used for image analysis and then wavelet reconstruction algorithm is used for image reconstruction. Image processing is done to give a better knowledge and understanding of the image by human or machine.  Figure 2 shows a general digital processing system.

This method requires the observer to make a reasonable evaluation of the restored image based on the judging criteria and the experience of the observer, so that the image closest to the human body is selected. Therefore, the corresponding gray level of the output image can be obtained using the following equation:

(3) $$\begin{array}{c} s_{k}=\sum_{j=0}^{k}p\left(r_{j}\right)=\sum_{j=0}^{k}\frac{n_{j}}{N},\;k=1,2,\ldots ,300,\\ g_{k}=\frac{s_{k}\times 300}{n+0.5}. \end{array}$$

*g*_*k*_—Gray scale value after gray scale transformation.

Since the memory-mapped file technique provided by the BSCB model can well solve the problem of handling large data files, the memory-mapped file method is used to map the park image and then recover the image when the recovery algorithm is actually implemented [28]. In order to make the recovery effect clear and avoid the intersection of iso-illumination lines, the BSCB model uses anisotropic diffusion to keep the edges smooth, and the recovery process and diffusion process are performed alternately. The block to be restored with high confidence value is usually restored first so that the restoration process is more reliable. The confidence is defined as:

(4) $$\begin{array}{c} C\left(p\right)=\frac{\sum_{q\in \psi_{p}\cap \varphi }C\left(q\right)}{\left|\psi_{p}\right|}. \end{array}$$

*C*(*p*)—Confidence level, |*ψ*_*p*_|—Area of *ψ*_*p*_.

Secondly, the whole gray value is divided into several straight lines, the desired image details are refined, the contrast is improved, and the excess details are compressed. Image properties are attributes that can be used as markers and can be generally classified into two categories: one is image statistical properties and the other is image visual properties [29]. Point operations are mainly addition, subtraction, multiplication, and division of object elements [30]. The iterative recovery method of wavelet transform requires more transformation operations and occupies more memory when recovering images. Therefore, the most optimal estimation error square is

(5) $$\begin{array}{c} p_{0}=A^{T}P\bar{A}={\left(e\bar{T}P^{-1}e\right)}^{-1}, \end{array}$$

*A*^*T*^—Weighted matrix; $\bar{A}$—Average weighting matrix.

Therefore, the observer of the recovered image needs to have some observation experience and a clear evaluation guideline before observation so that the observer can give an appropriate score after careful observation. By performing point operations on the image, the histogram distribution of the image can be effectively changed so that the clarity and uniformity of the image can be improved.

Finally, the grayscale of the output pixel is determined by the specific relationship of the grayscale of the input pixel, without changing the spatial relationships within the image. In fact, providing the desired reference image is frequently impossible. An objective image quality assessment method without reference can be used in this case. Image comprehension is a type of data derived from associating, thinking about, and comprehending an image's content. That is, the location of the file on your hard disc that corresponds to an identical area within your processing sequence's logical address space. The differences between areas in an image are based on the image's characteristics in different areas, but similar area properties exist within the same area. This correspondence is only a logical concept because there are no entities in the logical address space. The file is not loaded into memory during memory mapping, and no real copy of the data is created; only the data structure related to the initialization is created.

### 3.2. Histogram Transformation in Restoration of Long March Park Images

Most of the Long March cultural relics are distributed in poor areas and ethnic areas. Due to various factors such as geographical location, traffic condition, management difficulty, and financial investment, they cannot be restored and protected in time, and only some simple temporary maintenance can be carried out. Histogram correction is another kind of contrast enhancement based on probability theory, which converts the gray level of an image. The objective evaluation criteria of image quality mainly include peak signal-to-noise ratio and minimum mean square deviation, and these two indexes are selected as the main evaluation criteria:

(6) $$\begin{array}{c} \text{MSE}=\frac{\sum_{x=1}^{M}\sum_{y=1}^{N}\left[I_{0}\left(x,y\right)-I_{1}\left(x,y\right)\right]}{M\times N},\\ \text{SNR}=10\times \mathrm{lg}\left[\frac{\sum_{x=1}^{M}\sum_{y=1}^{N}\left[I_{0}{\left(x,y\right)}^{2}\right]}{\sum_{x=1}^{M}\sum_{y=1}^{N}{\left[I_{0}\left(x,y\right)-I_{1}\left(x,y\right)\right]}^{2}}\right]. \end{array}$$

At present, the Long March scenery is dominated by venues, monuments, and memorial squares, and tourist attractions are operated by field trips, picture displays, and text displays. In this way, the more evenly the image is distributed in the histogram, the more information is available and the clearer the image is. The histogram equalization technique is used to make the image constant in the number of pixels in a certain gray area by redistributing the pixels in the gray area, while the histogram basically follows the Hooke distribution.  Figure 3 shows a wavelet analysis for images.

First, for a particular image to be processed, if for each gray value, we count the number of pixels of that gray value. Sampling samples are shown as squares superimposed on a function. However, the sampled values of these gray levels at discrete locations, i.e., functions, are usually continuous. For this reason, a sequential iterative recursive calculation of the basic equations of the Kalman filter allows the calculation of the optimal estimate of the state at the *k* moment of interest. The weighted least squares estimation expression is

(7) $$\begin{array}{c} x=\arg\min\frac{1}{N}{\left(Z-CX\right)}^{T}W\left(Z-C\bar{X}\right). \end{array}$$

*W*—Weighted matrix.

Due to the random motion of the particles loaded during image acquisition, the image is noisy. External electromagnetic waves, for example, may cause interference with the imaging system. It creates noise in the environment. As a result, following memory mapping, a pointer to an address in the process's logical address space is obtained, which is then used to process the file. This method is simple to use while still preserving image edge information. However, if the damaged area is larger than the target structure's width, the visual connectivity principle cannot be applied, and if the slope is not steep enough, steps may occur. To reduce the computational process and speed up the computation, normalisation and minimization of the rise and fall function should be used when solving the partial differential equation. To achieve image tracking, the method uses the image's pixel position information to determine the center of mass of each colour block. To calculate the center of mass of each color cell *i*.

(8) $$\begin{array}{c} K_{i}^{n}=\frac{\sum_{i=1}^{n_{h}}\delta \left[b\left(X_{i}\right)-u\right]X_{i}}{\sum_{i=1}^{n_{h}}\delta \left[b\left(X_{i}\right)-u\right]}. \end{array}$$

*n*—*n* frame image, *X*_*i*_—Pixel position in the target area, *μ*—Histogram color value, *b*(*X*_*i*_)—Color value of pixel.

Secondly, a grayscale map of the pixels is drawn using the grayscale values and the corresponding number of pixels, which is called a grayscale map. At the same time, the method converts various a priori information in the segmented image into local features. The so-called scattering means that the leveling parameters are continuously changed in the wavelet, so that the leveling parameters are still varied by discrete in the time domain. Discretization of the grayscale is also required to obtain the numerical function. MMU is unable to find the entity address corresponding to this address mapping table when processing the archival information, and therefore a missing page interrupt occurs. The response function of the page break interrupt looks up the corresponding page in the virtual memory.

Based on this, the grayscale histogram of the original image is distributed equally from the more dense areas to different areas. The quantization of the image is achieved by comparing each sample gray scale with 8 discrete gray scales, and then using the most similar discrete gray scale as the gray scale. The gray value of the pixel itself is a common characteristic of the pixel. In color images, statistical features, texture features, and light intensity values of red, green, and blue colors can be used as feature characteristics. Since it is difficult for the current PC algorithm to correspond the high-resolution remote sensing image to the process address space at one time, and the amount of data mapped to the process address space cannot be larger than 1.5 GB each time.

## 4. Application and Analysis of Wavelet Transform Image Enhancement Algorithm in Image Restoration of Long March Park

### 4.1. Analysis of Filtering Colored Noise in Wavelet Domain

A wavelet is actually a function that is defined only within a certain range, beyond which it is almost zero. Noise in an image can be understood as “interference with the understanding and analysis of the received image information.” To obtain a simulated image, the image is wavelet transformed and processed with color noise. Then, we use the *P*-Laplace method to correct the wavelet coefficients for different loss rates. This is shown in Figure 4.

First, we expand the function to be close to zero and give it a set of functions. The distribution coefficients of wavelets and noise are diametrically opposed, and the coherence of the coefficients in wavelet space is small. Wavelet coefficients can be divided into two types. One has more signal and smaller amplitude after noise processing. The second path comes from multiple transformations. The original image is decomposed at different resolutions and then divided into different levels, which are then reconstructed. The cross-regional cooperation between “image restoration” and “Long March National Park” is not only the concept of “park,” but also the purpose and policy of “park” construction. It is not only the concept of “park” but also the purpose and policy of “park” construction. It is numerically simulated by parameters such as curvature and slope. In the curvature of a large area, the curvature of a small area has a stronger propagation ability. It uses balancing and correction techniques to average gray areas to the original image. As the gray level increases and the average value increases, the contrast increases, resulting in sharper details in the image. The low frequency coefficients of the first and second layers are recovered using wavelet recovery techniques, and the high frequency coefficients of each layer are obtained by a histogram matching operation. The three-level grayscale conversion curve is shown in Figure 5.

Secondly, the signal is extended to obtain the low frequency characteristics of the signal; the disadvantages of wavelet filtering are Gibbs effect and unclear boundary. In order to solve this problem, an invariant wavelet transform method is proposed in this paper. And the numerical simulation is carried out by applying the finite difference method. When the wavelet coefficients exceed the threshold value, the wavelet coefficients are set as wavelets. Waves lower than this threshold will be excluded. Based on the recovery of the isochronous region, each block of images is combined with it to achieve the recovery purpose. The selected threshold filter needs to have a high regularity. The change of polynomial filter factor using sub-segmented polynomials at 5, 10, and 15 times is shown in Figure 6.

Finally, the signal is processed using the systolic function in order to extract the signal's high frequency information. A better image enhancement effect can be achieved if the noise, edges, and other parts of the signal can be distinguished and processed separately. An adaptive image enhancement method is proposed for this purpose, which improves the enhancement effect by adjusting the adjustment factor based on the image's neighbourhood characteristics. The route direction and spatial boundaries of the Long March are scientifically determined, more complete Long March relics, stories, and memories are excavated, restored, and linked, the park's integrated development is accelerated to promote identity, and the integrity protection and authenticity inheritance of Long March relics and resources are promoted through regional cooperation. As a result, the generalized minimum problem is transformed to the wavelet domain and solved using an iterative method. While the CCD acquires digital images and the PSF in image processing is quantitative, the variation of PSF in a real imaging system should be continuous. The restoration model's discrete format is then given, and the damaged image is repaired to obtain the restored image.

### 4.2. Analysis of Improved Image Restoration Algorithm Based on Wavelet Transform

In the wavelet domain, the image is decomposed according to the image recovery model by minimizing a variational generalized function about the variables, i.e., solving for the extremes of the generalized function, which is the core problem of the variational method. As a linear tourist destination, the national cultural park faces many realistic problems due to its large spatial and temporal span, complex regional culture, and obvious boundary barriers. Therefore, it is particularly important to analyze the improved wavelet transform-based image recovery algorithm.

First, the wavelet coefficient sequence of the recovered part of the image is obtained by solving the generalized minimal value of Aujol, and the limit of the reconstructed sequence is obtained as the recovered part of the image. However, the loss of wavelet coefficients leads to inhomogeneity of the damaged area in the pixel domain, which makes the restoration theory of wavelet domain different from the traditional image domain restoration. The series of scale spaces formed by stretching or compressing the same scale function by the translation sequence have inclusion relationship, and their mutual inclusion relationship is shown in Figure 7.

Unlike the Great Wall and the Grand Canal, which are mainly “flow lines” and lack overall features, it is not only difficult to recover, but also not conducive to the recovery of the overall plan. In practical applications, image segmentation and reconstruction using low wave thresholds requires a high parametric regularity. Rotate the horizontal template around the center of the template to obtain filters in each direction. The corresponding filters are selected to perform directional filtering within a certain range.

Next, point operations are performed on the image in the spatial domain to change the grayscale of the pixel on the image to obtain a new image, and then point operations are performed. The image recovery uses the minimum energy equation. First, by searching the names of 166 tourism sites directly related to tourism resources, the corresponding keyword database was initially established through comparison and screening. On this basis, the orthogonal method was used to perform simultaneous orthogonal diffusion in the slope and slope directions, so that the damage area could be filled effectively. In the direction perpendicular to the ridge, the template coefficients were positive in the middle and negative on both sides. Then, PSNR was used for image restoration, and the similarity between *P*-Laplace and wavelet transform was compared, as shown in Tables 1 and 2.

The comparison shows that the algorithm in this paper has an average reduction of 223 in the number of iteration steps and an average improvement of 11.264 in the signal-to-noise ratio than *P*-Laplace, so a higher peak signal-to-noise ratio can be achieved with fewer iteration steps, especially in the case of high loss rate of wavelet coefficients.

Finally, the contrast of the structures of interest in the image is amplified to increase intelligibility; or the blending noise in the image is reduced or suppressed to improve the visual quality. In some cases, the image to be fused contains a large amount of redundant information, and the above fusion methods can yield richer information for cases where the source images do not differ much. However, at the same time, the edges and contours of the images tend to be blurred to some extent and the contrast of the images is reduced. Therefore, a segmented linear method is used to divide the gray value interval into several line segments, stretching the desired image details, enhancing the contrast, and compressing the unwanted details. The contrast before and after linear grayscale transformation is shown in Figure 8.

The curvature is introduced into the *P*-harmonic model so that it is related to curvature, gradient, and other factors. The small curvature region with large curvature has a stronger propagation ability. The curvature and *P*-Harmonic represent the aggregation and radiation functions of individual nodes in a directed traffic network. The number of strata indicates the importance of each service node in the network, while the modular network is divided into small regions of interest for each. After filtering, it is found that the regions which are more different from the surrounding areas have lower grayscale and are similar to the surrounding areas. With the Long March Memorial Hall as the carrier, the important meeting places, important battle sites, and iconic attractions along the Long March are reproduced. Make the red tourism brand of the Long March theme become an important position to inherit and carry forward the spirit of the Long March, cultivate and practice socialist core values, and a vivid window to promote new achievements in tourism and economic and social development along the Long March.

## 5. Conclusions

The Long March National Cultural Park is a new platform and a way to promote and carry forward the cultural heritage of the Long March. In today's world of deepening cultural tourism integration and increasingly refined cultural tourism consumption, the success of cultural tourism is crucial. It is very realistic and practical to promote the spirit of the “Thousand Mile Long March,” enhance the unique spiritual identity of the Chinese nation, strengthen the “fourfold self-confidence,” and fully demonstrate China's beautiful landscape, long history, and colorful national culture. Image degradation recovery is a theoretical and practical science. The high-resolution, time- and frequency-localized features of wavelet analysis make wavelet transform recovery more effective. In this paper, the wavelet transform is improved with wavelet domain color noise, and the enhancement of Long March Park image is combined with wavelet transform principle. After obtaining the histogram of the original image, an image fusion method is used to combine the uniform low-frequency subgraph and histogram to obtain the final enhancement effect. The wavelet transform-based image enhancement method, based on the wavelet transform technique, analyzes and fuses different images by the similarities and differences of the same image to achieve the recovery of that image.

## Figures and Tables

**Figure 1:** Block diagram of image fusion denoising based on wavelet transform.

**Figure 2:** Basic structure of digital image processing system.

**Figure 3:** Image restoration process based on wavelet transform image enhancement algorithm.

**Figure 4:** Comparison of PSNR between two algorithms after image restoration.

**Figure 5:** Transformation curves of gray values of three different layers.

**Figure 6:** Changes of polynomial filter factors with different segmentation times.

**Figure 7:** Projections of continuous signals at different scales.

**Figure 8:** Contrast before and after piecewise linear gray scale transformation.

**Table 1:** Comparison of peak signal-to-noise ratio after restoration by two algorithms.

	Loss rate	10%	20%	30%

PSNR/dB	*P*-Laplace	38.243	41.276	48.364
	Algorithms in this chapter	45.265	54.293	62.119

**Table 2:** Comparison of iteration steps between two algorithms after repair.

	Loss rate	10%	20%	30%

Iterative steps	*P*-Laplace	249	563	768
	Algorithms in this chapter	113	352	476

## Data Availability

The data used to support the findings of this study are available from the corresponding author upon request.
